The article "An Automated Deep Learning Model for the Cerebellum Segmentation from Fetal Brain Images" was retracted in 2023. Reasons: signs of a paper mill; suspected computer-generated content; unreliable results or conclusions; concerns about the data.

# An Automated Deep Learning Model for the Cerebellum Segmentation from Fetal Brain Images

**DOI:** 10.1155/2022/8342767

**Published:** 2022-06-16

**Authors:** R. Sreelakshmy, Anita Titus, N. Sasirekha, E. Logashanmugam, R. Benazir Begam, G. Ramkumar, Raja Raju

**Affiliations:** ^1^Department of Electronics and Communication Engineering, Veltech Rangarajan Dr Sagunthala R&D Institute of Science and Technology, Avadi, Chennai, 600062 Tamil Nadu, India; ^2^Department of Electronics and Communication Engineering, Jeppiaar Engineering College, Semmenchery, Raghiv Gandhi Salai, OMR, Jeppiaar Nagar, Chennai 600119, India; ^3^Department of Electronics and Communication Engineering, Sona College of Technology, Salem, 636005 Tamil Nadu, India; ^4^Department of Electronics and Communication Engineering, Sathyabama Institute of Science and Technology, Chennai, 600119 Tamil Nadu, India; ^5^Department of Electronics and Communication Engineering, Rajalakshmi Engineering College, Chennai, 602105 Tamil Nadu, India; ^6^Department of Electronics and Communication Engineering, Saveetha School of Engineering, SIMATS, Chennai, 602 105 Tamil Nadu, India; ^7^Department of Mechanical Engineering, St. Joseph College of Engineering and Technology, St. Joseph University, Tanzania

## Abstract

Cerebellum measures taken from routinely obtained ultrasound (US) images have been frequently employed to determine gestational age and identify developing central nervous system's anatomical abnormalities. Standardized cerebellar assessments from large-scale clinical datasets are required to investigate correlations between the growing cerebellum and postnatal neurodevelopmental results. These studies could uncover structural abnormalities that could be employed as indicators to forecast neurodevelopmental and growth consequences. To achieve this, higher-throughput, precise, and impartial measures must be used to replace the existing human, semiautomatic, and advanced algorithms, which seem to be time-consuming and inaccurate. In this article, we presented an innovative deep learning (DL) technique for automatic fetal cerebellum segmentation from 2-dimensional (2D) US brain images. We present ReU-Net, a semantic segmentation network tailored to the anatomy of the fetal cerebellum. Moreover, we use U-Net as a foundation models with the incorporation of residual blocks and Wiener filter over the last 2 layers to segregate the cerebellum (c) from the noisy US data. 590 images for training and 150 images for testing were taken; also, we employed a 5-fold cross-assessment method. Our ReU-Net scored 91%, 92%, 25.42, 98%, 92%, and 94% for Dice Score Coefficient (DSC), F1-score, Hausdorff Distance (HD), accuracy, recall, and precision, correspondingly. The suggested method outperforms the other U-Net predicated techniques by a quantitatively significant margin (*p* 0.001). Our presented approach can be used to allow high bandwidth imaging techniques in medical study fetal US images as well as biometric evaluation on a broader scale in fetal US images.

## 1. Introduction

Higher-frequency sound waves are used in the US imaging method to provide visible images of interior organs, blood flow, and tissues. It would be the most common method of fetal monitoring throughout pregnancy. It is usually utilized for vascular, thyroid, and abdominal scans, and it is rarely utilized to image air-filled tissues or bones like the lungs. The US imaging usage benefits are radiation-free and quick. Fetal brains in ultrasound (US) imaging had helped doctors better understand normal fetal brain growth and pinpoint brain anomalies in high-risk fetuses. Numerous subcortical regions in the fetal brains are examined with ultrasound (US) imaging during pregnancy. The US laser can pierce the fetal skull and visualize the subcortical structures, particularly early in pregnancy when the fetal skull has not entirely calcified. The subcortical structure abnormal development can be a possible symptom of a serious neurological illness, and as being such, it is essential to track their growth during pregnancy. With focused prenatal neurosonography, brain development could be investigated in great detail [1]. This will only be done in fetuses at higher risk for CNS disorders that is not part of the standard obstetric evaluations. The midbrain, cerebrum, cerebellum, and thalamus are all measured on US imaging as component of the fetal abnormality screening that takes place between 18 and 21 weeks of pregnancy. Modifications in cerebellar growth have been associated to neurodevelopmental abnormalities in overall mental development, motor function, and illnesses like autism, according to research [2, 3]. In fetal's embryonic stages, the cerebellum has been largely preserved, clearly differentiated from adjoining brain structures, and thus straightforward to examine on regular US scans. As a result, the cerebellum would be an important objective structure for researchers looking to better understand neurodevelopmental results and uncover prenatal perturbations that alter its growth. Semiautomatic or manual procedures are currently used in clinical practise to measure the cerebellum from the US imaging. Semiautomatic approaches need user input to set the cerebellums “end points” that are employed through an automated method to create assessments, while manual measures need free-hand interpretation by an experienced practitioner. However, both of these procedures have consumed more time and demand significant clinical competence, as they involve nuanced estimations of the cerebellar width from US pictures of varied sizes according on the fetus' appearances. Motion distortions, signal dropout, and nonuniform color clarity are also prevalent in US visuals. As a result, steps needed be taken to create analysis approaches that can enhance subcortical evaluation during regular gestation monitoring. Because of weak soft tissue differentiation, reverberation aberrations, and the typical occurrence of speckle make anatomical segmentation in fetal brain, US has been a difficult process. As a result, it might be difficult to detect specific structural limits, resulting in considerable intra- and interobserver heterogeneity in manual observations. Even experienced ultrasonographers may have difficulties in effectively segmenting thalamic regions in 3D US data because human segmentation would not be a procedure commonly undertaken in clinical practise. The fetal brain's fluctuating position because of the uncertain fetal position in the womb, and also transducer relative movement to the fetal head, is an US data additional issue taken with a free-hand screening approach, as is customary somewhere at bedside.

Deep learning (DL) algorithms have recently been proven to be effective in performing various segmentation operations in 3D US images of the fetal brain [4–6], outperforming classic image analytical techniques. Moreover, due to the challenges of getting manual labels for subcortical structures, attaining required ground-truth labels for training is a major hurdle to using DL techniques to this work. Few-shot learning could be employed to avoid the need for a huge manually labeled dataset by using only very few number of hand inputs, convolutional neural network (CNN) has been trained. Numerous few-shot learning techniques for segmentation purpose in the clinical image domain were developed [7, 8], demonstrating that high segmentation results can be enhanced with very little voxel-wise human annotation. We will employ a different DL-based approach for segmenting numerous brain structures in 3D US in this paper. Few-shot learning was not used for this purpose towards the best of our understanding.

## 2. Deep Learning (DL) overview

### 2.1. DL-Based Classifier (DLC)

DLC may directly process raw images, eliminating the requirement for preprocessing, segmentation, and extraction of features. Due of the input value constraint, most DL algorithms need image scaling. Although some approaches necessitate intensity normalisation and contrast adjustment, they can be prevented if data augmentation approaches are utilized during the data training. As a consequence, DLC seems to have a greater classification accuracy since it may prevent errors caused by an incorrect feature vector or inaccurate segmentation [9]. The research focus has changed from conventional image processing methods for future engineering to design of network architecture for optimized performance, due to DLC-based methodologies. DLC networks often include numerous hidden layers that means the algorithms seem to be more computationally expensive than ML-based techniques because more mathematical process is performed. The feature vector has been the input to the ML classifier, and the outcome is the object category, whereas the image was given as input to the DL classifier, and the result is the object category. DL might theoretically be considered an enhancement over traditional artificial neural networks (ANN) because it has many layers than the ANN [10]. Every layer translates the input image from the preceding layer into a compact representation at a greater and slightly greater level of abstraction, making it as representational type learning [11]. As a result, the model may acquire entire datasets both inter- and local-relationships in a hierarchical system. A nonlinear-based function is used to translate data into representations in DL models each layer. Generally, features derived from a particular image's initial layer of depiction will detect the existence or lack of edges in particular alignments, as well as their position in the picture. The secondary layer identifies patterns by recognizing disregarding small variations and edge positioning in these locations, whereas the third layer categorizes these structures into larger combinations that correspond to similar object fragments, allowing subsequent layers to identify objects using these configurations [10].

### 2.2. DL Architecture: CNN

CNN has been the most extensively employed DL architecture since it is fairly comparable to traditional NN. CNN receives an input as images, and it has a tri-dimensional network of neurons, which link to preceding layer's small region rather than the complete layer. A nonlinear activation layer like the pooling layer, Rectified Linear Unit layer (ReLU), or fully connected layers and convolutional layer is the CNN layers. The convolutional layer performs a convolution among input picture pixels and a filtration to generate feature map volumes containing features retrieved by the filters. ReLU seems to be a nonlinear activating layer, which employs a variable *f*(*x*) = max(0, *x*)  to input data to boost training speed and nonlinearity. Because the calculations are dependent on surrounding pixels, the pooling layers off the input data to mitigate the image spatial dimensionality to minimize computing cost and avoid overfitting [12]. Moreover, the CNN's last layer is fully connected layer, and it works similarly to hidden units in classic NN in which all neurons inside this layer have been interconnected to previous layer neurons. As previously stated, CNN is commonly employed to solve categorization difficulties. The input image is separated into small sections of identical size to employ CNN for semantic-based segmentation. Further, the patch's central pixel is classified by the CNN. The patches are then advanced to the next centre pixel to be classified. However, because the sliding patches overlapping features have not been reused, the image's spatial data is missing when the features migrate into the ultimate fully linked network layers. To address this issue, a fully convolutional network (FCN) has been presented, wherein the CNN's fully connected layers were replaced with transcribed convolutional layers, which apply upsampling in less-resolution feature space to retrieve the original spatial size even as trying to perform semantic segmentation [13]. Deep neural networks (DNN) are generally trained by combining the back-propagation technique with an optimization technique such as gradient descent. The procedure entails determining the loss function's gradient, which the optimization technique uses to modify the network weights in order to minimize the loss fitness values.

### 2.3. Other Architectures

#### 2.3.1. Autoencoder-Based DL Designs

An autoencoder NN seems to be an unsupervised-based learning method that generates the back-propagation technique with predicted values that are similar as the inputs to compact the input data into a series of hidden layers. It is divided into two parts: (1) the encoder, which compresses the input images into a series of hidden layers represented by function; *h* = *f*(*x*), and (2) the decoder, which recreates the input images from the series of hidden layers. The compressing is accomplished by limiting the hidden layer's size to those of the input nodes. Undercomplete networks are such networks. The hidden layer's reduced dimensionality causes the network to know the most important features inside the training set. A sparsity limitation, on the other hand, can be used to obtain comparable effects by maintaining hidden layer neurons inactive for the majority of time. The picture is subsampled to generate a lower dimension latent representation, allowing the autoencoder to be learned and operate on the image compact form in autoencoder-based deep learning systems.

One of the difficulties with autoencoders would be that the hidden layer's number of nodes exceeds the number of given input values. The concern is that the network will acquire a blank or identical function, where the output matches the input. To address this problem, denoising autoencoders have been employed to purposefully corrupt data by allocating input values about 30–50% to zero at arbitrary. The number of nodes within the network and the quantity of the information determine the real values lowered to zero. The outcome is compared to the actual input while generating the loss function, which eliminates the null function learning risks. Autoencoders have restricted applicability due to discontinuity in latent space interpretations that prevent them from being used as generative models. Thus, variational autoencoders have been developed to address this problem. In the variational autoencoder, encoder output is not a solitary encoded vector but dual encoded vectors: one is mean vector, while the other is the standard deviation vector. Those vectors serve as variables for a random vector that is used to test the encoded vector's outputs. This enables the decoder to reliably interpret the encoded data even when the source is somewhat different throughout training. Because of the autoencoder's unpredictable character, the latent space layers are designed to be continuous, enabling for randomized sampling and interpolation.

#### 2.3.2. Generative Adversarial Networks (GANs)

The goal behind GANs is to provide generators built as a NN, which represents a transformation function that accepts a random parameter as inputs and so when training matches the specified distributions. The other network was concurrently trained like a determiner to differentiate between fabricated and actual data. These two networks compete against each other, with the first attempting to maximise the last classification error among produced and genuine information and another attempting to minimize it. As an outcome, with each repetition of the training phase, both networks were enhanced.

#### 2.3.3. Restricted Boltzmann Machines (RBM)

RBMs are NNs that are predicated on energy-based models (EBMs). By attributing scalar energies to variables each specific configuration, EBMs encode dependency among variables. The observable variable values are used to learn or forecast the residual variable values in order to minimize energy use. Learning is accomplished by establishing an energy functions, which produces low energy for correct residual parameter values and bigger energies for incorrect values. The loss function that is minimized during training is used to determine the various energy functions superiority. In RBM, there is no output layer. Moreover, RBM has one input layer, a bias vector, a weight vector, and one hidden layer. During RBM training, network variables that minimize the energy function have been calculated for certain inputs. The neuron value in the hidden and input layers suggests the condition at a certain point in time, and all these values denote whether the associated neuron is inactive (state 0) or active (state 1). Deep belief network (DBN) is a form of RBM created via stacking, whereby each layer interacts with the layers above and below it. Undirected interconnections are found in the first two layers, whereas directed linkages are found in the bottom levels. DBM, on the other hand, is a sort of RBM network that solely comprises undirected interconnections. In the noisy input presence, DBMs have been thought to determining factors better.

#### 2.3.4. DL Structures Based on Sparse Coding

Sparse coding seems to be a type of unsupervised learning in which the input information is held by an overfitted collection of basis functions. Overfitted implies that the hidden representation's size is greater than the inputs. The goal is to find this basis vector linear combination that corresponds to a specific input. Because the network is overfitting, extra sparsity constraints must be implemented to handle any decadence. Sparse coding has the benefit of detecting connections between comparable descriptors and capturing important visual features [12].

#### 2.3.5. Recurrent NNs (RNNs)

RNNs have been designed to process with series kind inputs while the input size cannot be predicted. Because the series input does have an effect on its nearby values, it differs from many other inputs, and the networks must identify this connection. RNNs were networks that produce current output depending on both present learning and input from previous values. The previous input data is kept in a hidden linear system as segment of the system. This implies that based on prior inputs inside the sequence, the similar input might produce different outputs. Whenever the network is modified with various input series values over and over again, it creates various fixed-size output vectors. To every input, the hidden value is refreshed. RNNs could be given extra complexity by introducing more layers among the output and the hidden state layers, additional nonlinear hidden units between the hidden state and the input layers, or hidden state layers, or by combining all three methods.

### 2.4. Common DL Architecture Implementation Methodologies

DL algorithms for image segmentation were used in a variety of ways. The NNs are trained from beginning in first method, which needs the huge labelled dataset availability and time-consuming to create and train. In the following step, the pretrained CNNs, such as AlexNet that has been trained to categorize 1.2 million greater-resolution pictures for 1000 various classes and is accessible via ImageNet Large Scale Visual Recognition Challenge 2010, could be employed [14]. In this strategy, the last several levels of the networks are often removed and replaced with modern task-specific layers. The networks for categorization of new images are implemented by combining the low-level characteristics acquired from million images in the initial layers with the operation-specific extracting features in the last layers. This has the benefit of saving time in execution because just a tiny number of weights must be determined. Transfer learning has been generally used with networks learned on ImageNet information and is superior to randomized weight initialization [15]. The third method involves using pretrained CNNs to retrieve features from raw data and then using those characteristics as inputs to construct a classical classifier such as a support vector machine (SVM) for categorization. The benefit of this strategy is that characteristics may be retrieved automatically for a huge amount of categorical variables, removing the requirement for time-consuming manual feature extraction.

U-Net, which was designed for segmenting biomedical image [16], and V-Net, which has been designed for segmenting voxel medical image [17], are two commonly known CNNs. A U-Net seems to be an FCN that has expansion and contraction path. Successive max-pooling and convolutional layers make up the contracting path. It is being employed to extract the features while keeping feature maps small. Convolutional and upconversion layers have been employed in the expansion path to regain the segmentation map size without losing location information. Localization information is shared from shrinkage layer to the extension layer via back-propagation. All of those are concurrent interconnections that allow signals to travel straight from one block to another block of network without requiring any further processing. Lastly, in the final segmentation outcome, the convolutional layer preceding the output transfers the feature representation to the requisite number of selected categories. V-Net was identical to U-Net in that it is divided into two parts: decompression and compression. The compression phase is divided into several stages, typically having 1–3 convolutional layers. The residue functional is trained at every level utilizing convolution process on volumetric information based on voxels. The compression method, like the pooling layer, uses convolution to lower the quality by 50%. The pooling layer, on the other hand, is not utilized to minimize memory usage. Parametric ReLU (PReLU) generally called as Leaky ReLU, which is a nonlinearity perceptron that is a generalisation of ReLU. The network's decompression section increases the feature map spatial support, resulting in enough data for voxel segmentation. To expand the inputs size, deconvolution is employed, and the residue functionality is trained in the same way as the network's compression section. The outcomes of feature maps from the convolution layers even before outcome are the equivalent size as the input matrix. The expected background and foreground location information contained in the 2 feature images. Skip connections have been employed in the same way as U-Net to pass location information from network's compression to the extension parts.

The key contribution of this research is described as follows:

1. Initially, fetal US brain image dataset is collected from the standard website Kaggle
2. Hereafter, a novel ReU-Net is developed and trained to the system for segmenting the cerebellum from fetal brain images
3. Then, the preprocessing function is performed to eliminate the errors and unwanted noise in the US brain images using Wiener filter
4. After this process, ReU-Net has been employed to train and segment the cerebrum
5. Moreover, the performance of proposed model is validated and evaluated regarding recall, precision, F1-score, Hausdorff Distance (HD), and accuracy

The rest of the paper structure is organised as follows: Section 2 describes the recent literatures related fetal brain image segmentation, Section 3 explains the materials used for study, and Section 4 describes the overall methodology of the presented model. Moreover, Section 5 describes the evaluation metrics used in this study, Section 6 describes the obtained results of the presented model, Section 7 explains the paper discussion, and Section 8 concludes the paper.

### 2.5. Related Works

Some of the recent literatures related to segmentation of fetus' cerebellum are described as follows:

Singh et al. [18] have presented a new DL technique for automated fetal cerebellum segmentation from 2-dimensional (2D) ultrasound images. ResU-Net-c, a semantic segmentation method tuned for fetal cerebellar anatomy, was also developed. Use U-Net as a basis framework with residual block (Res) incorporation and dilation convolution for cerebellum segmentation from noisy US images in this article. The researcher employed images for testing as 146 and training as 588; using 5-fold cross validation method The presented approach can be used to allow higher-throughput image processing in medical research fetal US images, as well as biometric evaluation on a broader scale in fetal US images. However, this approach does not automatically segment cerebellum from US brain images. Zhao et al. [19] have developed a DL–based automatic segmentation of fetal brain approach that outperforms atlas-based techniques in terms of accuracy and resilience. The Wilcoxon signed-rank method was used to assess the DL method's robustness with a 4D atlas-based segmentation technique on 65 normal fetus MR images. The suggested DL method for fetal brain segmentation is stable and robust, outperforming segmentation predicated on a 4D atlas, and also employed in research and clinical settings. However, the important evaluation metrics are not evaluated.

Hesse et al. [20] created a CNN for cavum septum pellucidum et vergae (CSPV), lateral posterior ventricle horns (LPVH), cerebellum (CB), and choroid plexus (CP) automatic segmentation from 3D US images. With just a few manual observations, segmentation efficiency that is near to intraobserver heterogeneity can be achieved. Lastly, the trained frameworks were implemented to huge US image segments from a broad, healthy population, yielding new US-particular growth curves for the various designs during the pregnancy's second trimester. Moreover, the accuracy of segmentation needs improvement. Fidon et al. [21] have demonstrated that the nnU-Net DL pipeline has difficulty generalising to new anomalous situations. To address this issue, the researcher recommended training a deep NN to reduce the per-volume loss distribution percentile over the full dataset. Moreover, this can be accomplished via distributionally robust optimization (DRO), according to the findings. DRO reweights the lower-performing training data, enabling nnU-Net to operate more reliably in all circumstances. Further, the segmentation process may take more time to complete.

Kim et al. [22] have developed a DL-based approach for calculating biparietal diameter (BPD) and head circumference (HC) with excellent reliability and accuracy. By distinguishing tissue image structures with regard to the ultrasonic propagation path, the suggested approach efficiently determines the head border. The proposed approach was evaluated on 70 US images after being trained on 102 labelled data sets. The findings revealed that the proposed model was more accurate. However, the developed model is evaluated on smaller datasets. Khalili et al. [23] proposed performing segmentation by CNN that uses images with synthetically created contrast enhancement as data augmentation to eliminate intensity inhomogeneity in a preprocessing phase to segmentation. The intracranial size is first extracted using a CNN. These findings show that the suggested method might potentially substitute or augment preprocessing processes like bias field adjustments, improving segmentation results. However, the developed model's error rate was not measured.

Avisdris et al. [24] have developed a fully automated approach for calculating the bone biparietal diameter (BBD), trans-cerebellum diameter (TCD), and cerebral biparietal diameter (CBD) from fetal brain MRI. The suggested automatic technique for calculating fetal brain biometric linear measurements from MR imaging performs at a manual level. It also has the ability to improve ordinary clinical practise by allowing for the measurement of fetal brain biometry in both normal and abnormal patients. However, the process takes more time for linear measurements. FaBiAN, a Fetal Brain MR Acquisition Numerical Phantom, was created by Dumast et al. [25] to recreate multiple realistic fetal brain's MR images together with their category labels. The analysis showed that these numerous synthetic labeled data, which were created for free and then reassembled using the targeted superresolution approach, can be employed to effectively domain adapt a DL system that segments 7 brain tissues. Overall, segmentation accuracy has improved dramatically, particularly in the deep grey matter, white matter, cortical grey matter, cerebellum, and brainstem. Moreover, this model is only applicable for smaller datasets.

Rackerseder et al. [26] presented a DeepVNet-based segmentation approach, evaluating the pretraining with modelled ultrasonic sweep combination to enhance automatic segmentation and allow entirely automatic registration initiation. In contrast to partial labels given as input, the qualitative evaluation suggests that along with pretraining, the networks can learn to generalise more as well as provide finer and more comprehensive segmentations. Venturini et al. [27] investigated the CNNs use for the numerous embryonic brain areas segmentation in 3D US images. Automated brain segmentation in fetal US images can follow brain growth during pregnancy and also provide useful data that can assist predict fetal healthcare results. Also, the researcher presented a multitask CNN for automatic segmentation of brainstem, thalamus, white matter, and cerebellar labels, which was provided by atlases. The methods provided here offer an intriguing proof of concept, demonstrating that the presented methodology can be used to solve the segmentation issues. However, the developed method is difficult to process. The overview of reviewed literatures is shown in Table 1.

## 3. Materials

The images were gathered from standard website Kaggle (https://www.kaggle.com/gokulappu04/fetalbrains) [28]. From the Kaggle website, fetal brain US images at 18-20 weeks were acquired. 740 2D fetal US pictures of the fetus trans-cerebellar region were acquired. A 5-fold cross-assessment was used in our research. Every fold employed 590 of the 740 photos for training and 150 for testing. TIFF files were used to create the images. To match the photos to the segmentation networks, we trimmed the images to 720 × 720 pixels and focused on the cerebellar region. The ground truth for the cerebellar area was created by a scientist under medical supervision and verified by doctors.

## 4. Proposed Method

### 4.1. U-Net

Ronneberger et al. [16] presented U-Net as a deep CNN for biomedical image semantic segmentation. Its goal is to assign a label category to every pixel in the images. U-Net enhances on the completely CNN model [29] by increasing the decoder module's capacity. A contraction path captures context, and a symmetrical extending path allows for exact localization in the design of U-Net.

### 4.2. Residual Network

Deep layers in CNN demonstrate that the layers learn more complicated features over time. This could be useful for discriminatingly learning the cerebellum's complicated visual features. Deeper networks, on the other hand, have larger testing and training error. Overfitting can be produced by the complex function constructions with more layers, according to He et al. [30]. This could explain why deeper networks collapse more often than shallower networks. With the application of regularisation settings and additional algorithm, the overfitting problem can be avoided. However, because of feature space's extensive exploration, the deeper network failures are also ascribed to the diminishing gradient problem. This renders it vulnerable to disturbances that could force it to depart the manifold and necessitate the acquisition of further labelled training data, which is tough to come by in the medical imaging field. RNN application has solved the training difficulty in a very deep network. Skip connections are used by the RNN to leap over some layers. Triple or double layer skips have been used in ResNet models. ReLU and normalisation of batch are commonly seen in these layers. By retaining weights learnt by an activation layer, the purpose for bypassing the layers is to reduce disappearing gradients. Furthermore, omitting layers in the training phases streamlines the network and eliminates the requirement for big training data.

Weights respond towards the mute upstream layer during training but also amplify the earlier ignored layer. The network eventually recovers the skipped layers as it acquires the feature space. While all layers were stretched towards the training end, it remains nearer to the manifolds, leading to rapid learning. With DNN, skip connections were proven to improve performance in a variety of image identification applications. We used hidden layers to boost the segmentation task performance in this work. The basic figure of residual block has been depicted in Figure 1. There are no variables in the identical mapping, but it is just employed to add the outcome from the prior layer towards the next layer. *F*(*u*) and *u* will not have the same sizes. To widen the skip channel to meet the sizes, the identical mapping is multiplied by (*V*_*z*_)  linear projection, which is shown in

(1) $$\begin{array}{c} w=F\left(u,\left\{V_{i}\right\}\right)+V_{z}u, \end{array}$$

where *F*(*u*, {*V*_*i*_}) indicates the residual mapping learning and *V*_*z*_ can implement the *n* convolutions. In this research, (1 × 1) Wiener filter was used in ReU-Net.

### 4.3. ReU-Net Architecture

ReU-Net accepts 720 × 720 pixels in size images as input and outputs a labeling image of the similar size. The networks have been separated into two sections: a left-hand encoder, which is contracting path, and a right-hand decoder, which is expanding path. There are six tiers in each path. The encoder module frequently lowers the input resolution, while the decoder component has difficulty in producing segmentations as fine-grained. Skip connections from previous layer allow fine layer information to be combined with rough layer characteristics, allowing ReU-Net to recognize the spatial structure during the segmentation process with fine-grain information. The remaining blocks were added to the networks to offer the features needed to recreate the shape of the cerebellum with proper boundaries.

The extended skip connections between the decoder and encoder modules matching feature maps have not been employed, apart from in typical U-Net design. We created brief hidden layers inside the blocks to enable quicker training intersections and deeper model training. Every residual block performs 2 kinds of Wiener filter procedures (1 × 1 and 3 × 3). To maintain the feature map size after the Wiener filter process, zero padding procedures are utilized. According to Singh et al. [18], the number of feature maps rises from minimum to maximum levels. The Wiener filter reduces the unwanted noise from US images. It concurrently removes the extra material noise and regulates the darkness. The filtering strategy is based on a stochastic architecture, and this form of filter is excellent regarding mean square error (MSE) [31]. The proposed method's workflow is shown in Figure 2.

In the projected ResU-Net design, to bring nonlinearity into the networks, ReLU has been employed as an activation function with all layers. Moreover, in the encoder component, max pooling with such a 2-pixel stride is employed from 1 to 3 layers. To reduce overfitting, this involves downsampling process along the spatial dimensions and decreases the amount of variables and calculations in the networks. It also aids in the input image representation being scale-invariant. In the decoding part, we employed upsampling levels to boost the feature map spatial resolution.

The output and input of upsampling and max pooling layers does not have a skip connection. The decoder and encoder blocks receive the upsampling and max pooling layer outputs, respectively. A solitary convolution layer having 1 × 1 kernel size makes up the forecasting layer. The label map was predicted using the Softmax layer. The presented method was implemented in Python and running on Windows 10 platform. Moreover, the network architecture of presented ReU-Net is shown in Figure 3.

### 4.4. Loss Functions

The discrepancy between the anticipated binary ground truth and binary output is measured and minimized using a loss function. The Binary Cross-Entropy (BCE), Dice Loss (DL), and the Focal Tversky Loss (FTL) were all employed. The segmented region overlap was measured using DSC, and the pixel wise concordance between the ground truth and output was measured using BCE. In training segmentation approaches, FTL was employed to tackle class imbalance concerns.

### 4.5. Dice Loss (DL)

The Dice Score Coefficient (DSC) seems to be an overlap statistic frequently often used that evaluates segmentation effectiveness in medical images. For category c, the two-class DSC variation is in

(2) $$\begin{array}{c} {\text{DSC}}_{c}=\frac{\sum_{i=1}^{n}P_{ic}g_{ic}+k}{\sum_{i=1}^{n}P_{ic}+g_{ic}+k}, \end{array}$$

where *g*_*ic*_ *ϵ* 0, 1 and *P*_*ic*_ *ϵ* 0, 1  represent the ground truth labeling and the anticipated label, correspondingly. The overall number of pixels in the image is denoted by *N*. To avoid dividing by zero, the *k* gives numerical stability. The final DL is described as the least overlap among the ground truth and prediction, which was given in

(3) $$\begin{array}{c} {\text{DL}}_{c}=\underset{c}{\sum }1-{\text{DSC}}_{c}. \end{array}$$

### 4.6. Combo Loss (CL)

DL and BCE loss were utilized in conjunction. The loss function of BCE can be written as below for two-class issues:

(4) BCEg,p=−1N∑gi.logpi+1−gi.log1−pi.i=1N

The CL is calculated as follows:

(5) $$\begin{array}{c} \text{CL}=0.5\times \text{BCE}+\text{DL}. \end{array}$$

For every loss, the CL is specified by a unique weight factor *w* *ϵ* [0, 1] [0, 1]. DL and BCE have *w* of 1 and 0.5, respectively.

### 4.7. Focal Tversky Loss (FTL)

To boost recall rate in a heavily unbalanced data set with a tiny background area, false negative (*F*_*n*_) observations must be rated greater than false positives (*F*_*p*_). Tversky resemblance index (TI) is a DSC scoring extension that provides for more versatility in harmonizing *F*_*n*_ and *F*_*p*_.

(6) $$\begin{array}{c} {\text{TI}}_{c}=\frac{\sum_{i=1}^{n}P_{ic}g_{ic}+k}{\sum_{i=1}^{n}P_{ic}g_{ic}+\alpha \;\sum_{i=1}^{n}P_{\bar{ic}}g_{ic}+\beta \sum_{i=1}^{n}P_{\bar{ic}}g_{ic}}. \end{array}$$

The chance that pixel *i* belongs to the category c cerebellum is represented by *P*_*ic*_, while the likelihood that pixel *i*  belongs to the background category c is represented by *P*_*ic*_. *g*_*ic*_ and $g_{\bar{ic}}$ have similar definitions. Whenever there is a big class unbalance, the hypervariables are adjusted to enhance recall. *β* = 0.7 and *α* = 0.3 were used in all of the studies. Moreover, TI loss is computed as follows:

(7) $$\begin{array}{c} {\text{FTL}}_{c}=\underset{c}{\sum }{\left(1-{\text{TL}}_{c}\right)}^{1/\gamma }. \end{array}$$

Here, *γ* is set as 4/3.

### 4.8. Training Parameters

In all of the simulations, the Grey-wolf optimizer was employed as the optimization technique. In all of the training trials, it performed better than other algorithms. The randomized weights have been used to set the model parameters; 1 × 10^−6^ was chosen as the learning rate. The training and validation datasets were split into two batches because of a high batch size, which slows the training.  Table 2 indicates the number of epochs and parameter training numbers employed in all the selected frameworks.

## 5. Evaluation Metrics

The fetal US brain segmentation system's effectiveness is assessed using conventional and well-known criteria, allowing for comparison with current methods available in the literature. The choice of a suitable evaluation measure is influenced by a number of aspects, including the system's functionality. Moreover, evaluation metrics are crucial in evaluating the segmentation model outcomes. We used F1-score, precision, accuracy, Hausdorff Distance (HD), and recall to evaluate our outcomes in this study.

### 5.1. Accuracy and Recall

Recall is the segmentation performance measures regarding under- and oversegmentation; here, low recall recommends under segmentation. True negative (*T*_*n*_) indicates a pixel, which is accurately identified as not being part of the ground truth. False negative (*F*_*n*_) indicates a pixel that was wrongly anticipated as ground truth. True positive (*T*_*p*_) indicates a pixel, which is accurately identified as ground truth, and false positive (*F*_*p*_) indicates a pixel, which was inaccurately identified as ground truth.

Recall is described as follows:

(8) $$\begin{array}{c} \text{Recall}=\frac{T_{p}}{T_{p}+F_{n}}. \end{array}$$

Accuracy describes the percentage of correctly segmented image pixels. Absolute pixel precision is another name for it. This is the most fundamental performance indicator, but it does have the potential to mislead picture segmentation results when there is a class mismatch. Whenever one segmented category exceeds another, category mismatch occurs. In this instance, the prevailing class' superior accuracy will outweigh other category's lower accuracy, resulting in skewed findings. If there is no group mismatch, the accuracy measure was suggested for measuring segmentation results with images. The accuracy of segmentation is calculated by

(9) $$\begin{array}{c} \text{Accuracy}=\frac{T_{p}+T_{n}}{T_{p}+F_{p}+T_{n}+F_{n}}. \end{array}$$

### 5.2. Precision and F1-Score

The fraction of cerebellum pixels in the automated segmentation outcomes that matches the ground truth cerebellum pixels is known as precision. Because precision is susceptible to oversegmentation, it is a relevant metric of segmentation results. Low precision values resulted from oversegmentation. The precision is computed as follows:

(10) $$\begin{array}{c} \text{Precision}=\frac{T_{p}}{T_{p}+F_{n}}. \end{array}$$

Recall and precision can be employed together because large values for both metrics for a certain segmented images indicate that the projected segmented regions matched the ground truth regarding location and detail level. The recall and precision's harmonic mean is determined by the F1-score, often referred as Boundary F1 (BF), which is helpful for boundary or contour matching between ground truth and predicted segmentation. F1-score is computed as follows:

(11) $$\begin{array}{c} \text{F}1–\text{score}=2\times \frac{\text{Recall}\times \text{Precision}}{\text{Recall}+\text{Precision}}. \end{array}$$

### 5.3. Hausdorff Distance (HD)

HD seems to be a segmentation error metric [32]. The level of proximity between two pictures is measured in HD. HD is calculated between the ground truth (*Q*) and predicted (*P*) segmentation borders, which are depicted as follows:

(12) $$\begin{array}{c} \text{HD }\left(P,Q\right)=\max\left(hd\left(P,Q\right),hd\left(P,Q\right)\right), \end{array}$$

where *h*(*P*, *Q*) = maxmin|*p* − *q*|; here, *p* *ϵ* *P*, and *q* *ϵ* *Q*.

## 6. Results

Table 3 indicates the performance of segmentation of the presented ReU-Net model with other models like U-Net++, U-Net, and Attention U-Net. The result indicated that the developed model has attained higher segmentation performance regarding precision, F1-score, recall, HD, and accuracy. Moreover, the processing time is also less than other methods. Thus, the developed method has higher efficiency than other models.

We contrasted ReU-Net to well-known segmentation approaches based on the U-Net architecture, like Attention U-Net [33], U-Net [16], ResU-Net-c [18], and U-Net++ [34]. We selected the DSC as the key assessment criterion for comparability while rating our models. The comparison result is shown in Table 4. SD represents standard deviation. The overall outcome of presented ReU-Net is shown in Figure 4.

## 7. Discussion

The ReU-Net recommended illustrates the usefulness of the remaining links in the U-Net format intended for US images. Along with the remaining volume, the low-level properties of the previous layers are fully integrated with the high-level properties of the recent layers, promoting the use of highly effective properties in cerebral separation. The importance of loss functions in establishing the performance of the network cannot be overstated. Table 3 shows the performance measurements for all comparative techniques with CL, TFL, and DL. In the remaining U-Net, DL performed much better, but the incorporated losses of BCE and DL performed better in other comparative techniques. Combining DL and BCE losses, the study looked at whether it would have distinct effects throughout the training phase. By upgrading the DL, the study found that CL activates the preferred trade between false positives and negatives and prevents entanglement in sublocal minima. Following training, CL integrates much faster than BCE. Although FTL has been found to be effective in severely unbalanced datasets, traditional loss operations appear to be more efficient.

According to research, FTL may not record ambiguities within the boundary. This creates separated mapping with better accuracy, but with less recall in practice. DL, on the other hand, has equal weights for FP and FN detection systems and improves performance in the recommended strategy. As a result, the performance of the losses process depends on the image features of curvature and random borders. The excellent accuracy of this method verifies the use of residual links and extended curves, making it highly suitable for dividing the cerebellum in US images. Research shows that this technique divides cerebellar structures most precisely than previous comparative methods. Due to the weak margins, the contours of the U-Net, U-Net++, and Attention U-Net model do not describe the exact parts of the cerebellum. Due to the lack of precise limits, they were affected by the leak and did not cover the entire area of interest. The recommended technique is the result of shattered outlines within the cerebellum, without the expansion layer. Other comparative approaches have revealed similar results, demonstrating the need for an expansion coil for cerebellar separation.

The recommended ReU-Net enhanced the visual effects on all models. With the DL feature, ReU-Net had the best DSC. The low accuracy of the comparison techniques suggests that there are a large number of noncerebellum pixels within the segmentation definitions. ReU-Net's enhanced accuracy reveals low FP in the expected cerebellum. When the HD scores of the recommended technique are compared with other modelling approaches, the recommended method is more statistically significant than the other comparison approaches (*p* 0.001). The researchers found that the image fragment performance was lower when the fetal head boundaries were not fully visible and/or there were pauses in all approaches. Anatomical visualization of the skull in the fetal head is one of the reasons for this poor performance. The study suggests that such images should be reversed from the automated processing of US images and instead evaluated for image quality.

ReU-Net works better than U-Net, but lower than recommended technique. The rich semantic information obtained through the skip links in the remaining volumes is credited with the enhanced performance of this technique. Without expanding the size of the network variables, the remaining practices dramatically increase training and testing performance. The results of ReU-Net were low on all scales, emphasizing the need to add expansion layers to the recommended technique. Wiener filters expand CNN's acceptance field without adding new variables, avoiding excessive matching problems during the training phase. The Wiener filter used in this technology allows the acceptance field to expand exponentially without losing spatial details. The learning curve for the recommended approach is steeper than previous approaches. Results of this magnitude show that the recommended approach to cerebral separation is accurate, robust, and reliable.

Manual cerebellum assessments are easy to make, and semiautomated procedures are quick; nevertheless, because these methods all rely on human inputs, their strength and stability are at risk. When a significant number of images are required, manual procedures can be time-consuming. The autoseparation approach allows for a retrospective research on a high quantity of US images. Image quality evaluation before the US film division of the automation nucleus will be part of future research. This technique will be extended to future cerebellar assessments and measurements in the future. The technique is believed to have the potential to reduce operator dependency in clinical applications for fetal health assessment, thus improving strength and reproducibility performance.

## 8. Conclusion

An intrusion detection approach through stacking dilated CNN is introduced and applied for recognizing as well as detects the attackers efficiently in wireless networks. Massive amounts of unlabeled original traffic data can be autonomously learned important feature representations using the suggested DL approach. The Contagio-CTU-UNB dataset and the CTU-UNB dataset were constructed using computer traffic data from different sources. To assess the proposed effectiveness of the algorithm, three different categorization activities are used. Deep learning method is compared to other techniques of a similar nature. The impacts of a number of vital hyperparameters are investigated further. Experiments show that the model outperforms others in detecting intruders from large amounts of data. By combining significant computational approaches, this method was able to accomplish exceptional performance that fulfils the demands of large-scale and real-world network systems.

## Figures and Tables

**Figure 1:** Residual block basic diagram.

**Figure 2:** Workflow.

**Figure 3:** Network architecture of ReU-Net.

**Figure 4:** Overall outcome of proposed ReU-Net model.

**Table 1:** Overview of reviewed literatures.

Authors	Reference	Year	Article title	Proposed approach	Type of images	Training images	Testing images	Limitation
Singh et al.	[18]	2021	2D fetal US brain images cerebellum semantic segmentation	ResU-Net-c	US	588	146	The model does not segment the cerebellum automatically
Zhao et al.	[19]	2022	Optimized DL method-based automated segmentation of 3D fetal brain images	3D U-Net	MR	65	41	Not all the evaluation metrics are computed
Hesse et al.	[20]	2022	Fetal brain's subcortical segmentation in 3D US images by DL methods	CNN	US	215	20	Segmentation robustness requires more improvement
Fidon et al.	[21]	2021	DRO-based abnormal brain of fetal segmentation using 3D MR images	nnU-Net-DRO	MR	116	26	The process of segmentation may take more time to complete
Kim et al.	[22]	2019	Fetal-head biometry automatic evaluation by ML	DL-based method	US	102	70	The method is employed only on smaller datasets
Khalili et al.	[23]	2019	Automatic segmentation of fetal brain tissue by CNN	CNN	MR	32	94	The error rate of developed method was not measured
Avisdris et al.	[24]	2021	Fetal brain automated linear measures by DNN	DNN	MR	121	33	The linear measurements take more time
Dumast et al.	[25]	2022	Segmentation of fetal brain tissue from synthetic MR images	FaBiaN	MR	17	11	The developed model is not applicable for large datasets
Rackerseder et al.	[26]	2019	3D brain US fully automatic segmentation	DeepVNet	US	N/A	N/A	The quantitative evaluation takes more time
Venturini et al.	[27]	2019	Structural semantic segmentation using multitask CNN from 3D US images	Multitask CNN	US	480	48	The presented approach is challenging

**Table 2:** Epochs and model parameter iteration.

Models	Epochs		Parameters
Attention U-Net	FTL	200	35,974,075
	DL	250	
	CL	150	

U-Net	FTL	200	32,842,032
	DL	250	
	CL	150	

U-Net++	FTL	300	11,284,042
	DL	150	
	CL	100	

ReU-Net (proposed)	FTL	120	18,742,832
	DL	127	
	CL	235	

**Table 3:** Segmentation fetal cerebellum evaluation.

Methods	Losing variable	Precision	Recall	DSC	F1-score	HD	Accuracy	*p* rate	Proceeding time (seconds)
Attention U-Net	FTL	0.84	0.79	0.84	0.85	40.05	0.92	4.20*E*-21	0.50
	CL	0.89	0.82	0.87	0.84	35.87	0.94	6.12*E*-87	0.45
	DL	0.86	0.85	0.82	0.88	34.25	0.91	5.24*E*-87	0.42

U-Net++	FTL	0.91	0.84	0.91	0.87	28.67	0.89	7.24*E*-65	0.35
	CL	0.89	0.87	0.89	0.82	25.50	0.85	4.20*E*-30	0.40
	DL	0.92	0.88	0.92	0.84	24.26	0.92	6.54*E*-40	0.32

U-Net	FTL	0.94	0.90	0.87	0.90	22.56	0.94	5.23*E*-01	0.30
	CL	0.91	0.92	0.88	0.91	30.02	0.92	3.20*E*-62	0.32
	DL	0.89	0.89	0.84	0.89	20.26	0.93	2.50*E*-64	0.38

ResU-Net-c	FTL	0.90	0.94	0.91	—	18.2	—	3.02*E*-01	0.32
	CL	0.95	0.9	0.91	—	17.8	—	9.52*E*-01	0.30
	DL	0.93	0.92	0.92	—	17.9	—	—	0.34

Proposed ReU-Net	FTL	0.94	0.95	0.94	0.92	18.24	0.97	4.50*E*-05	0.25
	CL	0.96	0.93	0.92	0.93	15.25	0.95	10.45*E*-21	0.20
	DL	0.94	0.92	0.93	0.94	15.78	0.98	—	0.23

**Table 4:** Fetal cerebellum segmentation by DL (i.e., mean ± SD).

Model	Precision	HD	Recall	*p* value	DSC
U-Net++	0.75 ± 0.24	42.12 ± 33.54	0.82 ± 0.15	5.42*E*-31	0.87 ± 0.18
Attention U-Net	0.85 ± 0.12	35.42 ± 28.52	0.72 ± 0.17	1.08*E*-27	0.82 ± 0.13
ResU-Net-c	0.92 ± 0.05	28.42 ± 27.6	0.74 ± 0.18	1.2*E*-38	0.88 ± 0.15
U-Net	0.82 ± 0.21	38.45 ± 21.5	0.82 ± 0.19	1.32*E*-23	0.74 ± 0.17
ReU-Net (proposed)	0.94 ± 0.07	25.42 ± 21.76	0.92 ± 0.18	—	0.91 ± 0.08

## Data Availability

The data used to support the findings of this study are included within the article.
